# Evaluation of Pt,Pd-Doped, NiO-Decorated, Single-Wall Carbon Nanotube-Ionic Liquid Carbon Paste Chemically Modified Electrode: An Ultrasensitive Anticancer Drug Sensor for the Determination of Daunorubicin in the Presence of Tamoxifen

This article has been retracted.

**DOI:** 10.3389/fchem.2020.00677

**Published:** 2020-08-19

**Authors:** Marzieh Alizadeh, Parviz Aberoomand Azar, Sayed Ahmad Mozaffari, Hassan Karimi-Maleh, Ali-Mohammad Tamaddon

**Affiliations:** ^1^Department of Chemistry, Science and Research Branch, Islamic Azad University, Tehran, Iran; ^2^Thin Layer and Nanotechnology Laboratory, Department of Chemical Technologies, Iranian Research Organization for Science and Technology (IROST), Tehran, Iran; ^3^Laboratory of Nanotechnology, Department of Chemical Engineering, Quchan University of Technology, Quchan, Iran; ^4^Center for Nanotechnology in Drug Delivery, School of Pharmacy, Shiraz University of Medical Sciences, Shiraz, Iran

**Keywords:** daunorubicin, tamoxifen, 1-butyl-2,3-dimethylimidazolium tetrafluoroborate, Pt,Pd-doped NiO nanoparticle, cancer sensor

## Abstract

Measuring the concentration of anticancer drugs in pharmacological and biological samples is a very useful solution to investigate the effectiveness of these drugs in the chemotherapy process. A Pt,Pd-doped, NiO-decorated SWCNTs (Pt,Pd-NiO/SWCNTs) nanocomposite was synthesized using a one-pot procedure and combining chemical precipitation and ultrasonic sonochemical methods and subsequently characterized by TEM and EDS analysis methods. The analyses results showed the high purity and good distribution of elements and the ~10-nm diameter of the Pt,Pd-NiO nanoparticle decorated on the surface of the SWCNTs with a diameter of about 20–30 nm. Using a combination of Pt,Pd-NiO/SWCNTs and 1-butyl-2,3-dimethylimidazolium tetrafluoroborate (1B23DTFB) in a carbon paste (CP) matrix, Pt,Pd-NiO/SWCNTs/1B23DTFB/CP was fabricated as a highly sensitive analytical tool for the electrochemical determination of daunorubicin in the concentration range of 0.008–350 μM with a detection limit of 3.0 nM. Compared to unmodified CP electrodes, the electro-oxidation process of daunorubicin has undergone significant improvements in current (about 9.8 times increasing in current) and potential (about 110 mV) decreasing in potential). It is noteworthy that the designed sensor can well measure daunorubicin in the presence of tamoxifen (two breast anticancer drugs with a ΔE = 315 mV. According to the real sample analysis data, the Pt,Pd-NiO/SWCNTs/1B23DTFB/CP has proved to be a promising methodology for the analysis and measuring of daunorubicin and tamoxifen in real (e.g., pharmaceutical) samples.

## Introduction

Cancer is a major disease known to be the leading cause of death in the world (Bernstein and Ross, 1993). It is estimated that more than 2.7 million cancer patients will be diagnosed worldwide by 2040, most of them suffering from one of the four main cancers (bowel, lung, prostate, and female breast) (Bernstein and Ross, 1993). Chemotherapy and the use of anticancer drugs are known as the mainstays of treatment for most cancers (Trichopoulos et al., 1972; Bernstein and Ross, 1993; Radwan et al., 2019). Therefore, much research is being done on the identification, efficacy, side effects, and effects of anticancer drug concentrations on the derma process and on the combined effect of anticancer drugs in the chemotherapy process (Delaney et al., 2005; Moseley et al., 2007; Andersen and Kehlet, 2011). Accordingly, research work in this area is of great importance for the global health sector (Moseley et al., 2007).

Daunorubicin in injectable form was introduced as a chemotherapy drug for different types of cancers, such as chronic and acute myelogenous leukemia and breast cancer (Skovsgaard, 1978; Slater et al., 1982; Raut, 2015). Daunorubicin, commonly prescribed in combination with other anticancer drugs in chemotherapy, such as tamoxifen, is used to reduce the side effects of surgery and the reinfection risk of breast cancer (Reiffers et al., 1996; Guo and Lu, 2010; Shien et al., 2014). Numerous studies have investigated the effects and benefits of the simultaneous use of daunorubicin and tamoxifen on the human body (Shao et al., 2012; Li et al., 2014). Therefore, this research has focused on the analysis of daunorubicin in the presence of tamoxifen.

There are different analytical strategies for the determination of daunorubicin separately or in the presence of other anticancer drugs (Hulhoven and Desager, 1977; Wang et al., 1987; Hu et al., 2000; Gavenda et al., 2001; Jiang et al., 2003). Electrochemical methods are attractive; fast, inexpensive, non-polluting analyses with good kit ability make such techniques more appealing than other analytical methods (Yuan et al., 2013, 2017, 2019, 2020; Fu et al., 2018, 2019a,b,c, 2020; Xu et al., 2018). However, the ability of electrochemical sensors to detect inappropriate levels is still limited due to the weak signal of pharmaceutical and biological compounds on the surface of unmodified sensors (Karimi-Maleh et al., 2017, 2020a,b; Ghanei-Motlagh and Baghayeri, 2020; Nodehi et al., 2020). With the replacement of simple sensors with electrochemical modified sensors in recent years, it has been possible to sensitively and selectively measure important drug compounds, especially anticancer drugs (Karimi-Maleh et al., 2019a; Khodadadi et al., 2019; Baghayeri et al., 2020; Karimi-Maleh and Arotiba, 2020; Mohanraj et al., 2020). Nanomaterials with new and wonderful features are important options in various fields in recent years (Rayati and Malekmohammadi, 2016; Asl, 2017; Malekmohammadi et al., 2018a,b; Orooji et al., 2019a,b,c; Karimi-Maleh et al., 2020c; Nguyen et al., 2020). Different types of nanomaterials have been synthesized and used as powerful materials in the recent years (Keyvanfard et al., 2014; Nayebi et al., 2016; Parvizi et al., 2018; Asl et al., 2020; Fattahi et al., 2020; Sakkaki et al., 2020). Metal-based nanomaterials, such as NiO, SiO, Au, TiO_2_, ZnO, Pt, and Pd showed high catalytic activity in different fields and especially electrochemical systems (Yang et al., 2010; Baghayeri et al., 2013, 2019; Mozaffari et al., 2014, 2015; Rahmanian and Mozaffari, 2015; Rahmanian et al., 2015; Asrami et al., 2017, 2018; Karimi-Maleh et al., 2019b, 2020d; Tahernejad-Javazmi et al., 2019). Recently, metal-doped metal oxide nanoparticles, such as the Pt-doped NiO nanoparticle were used as a high-performance electrocatalyst in fabrication of electrochemical sensors (Dehdashti and Babaei, 2020).

Ionic liquids are new conductive materials with excellent electrical conductivity that have garnered much attention and have been widely used as modifiers in the last 20 years (Atta et al., 2019; Shamsadin-Azad et al., 2019). Many researchers have demonstrated the separate or combined use of ionic liquids with nanomaterials to design electrochemical sensors (Alavi-Tabari et al., 2018; Beytur et al., 2018; Li et al., 2019).

According to studies and reviews of articles published in the field of electrochemical sensors, no research has been done on measuring daunorubicin in the presence of tamoxifen, and therefore, this project has undertaken the construction of an electrochemical sensor for this purpose. To that end, Pt,Pd-NiO/SWCNTs/1B23DTFB/CP was fabricated. The synergic effect of the Pt,Pd-NiO/SWCNTs nanocomposite and 1B23DTFB helped improve the ability of sensors to make highly sensitive determinations of daunorubicin under optimum conditions. In addition, this synergic effect created an interesting condition for determining daunorubicin in the presence of tamoxifen in real samples.

## Materials and Methods

### Instrumentation

The electrochemical part of this research was performed using an electrochemical workstation model Ivium-Vertex connected to an electrochemical cell (Azar Electrode Company, Iran). The TEM (made in Germany, model Zeiss-EM10C-100 kV) was used to characterize the Pt,Pd-NiO/SWCNTs nanocomposite. All recorded voltammograms are based on the Ag/AgCl/KCl_sat_ reference electrode (Azar Electrode Company) potential.

### Reagents

Daunorubicin, hydrochloride, sodium hydroxide, tamoxifen, 1-butyl-2,3-dimethylimidazolium tetrafluoroborate, and SWCNTs were bought from Sigma-Aldrich. Carbon powder, nickel nitrate hexahydrate, paraffin oil, phosphoric acid, and platinum(II) acetylacetonate were bought from Merck Company. 0.001 M stock solutions of daunorubicin, hydrochloride, and tamoxifen were prepared in 100 mL distillated water by dissolving 0.56 and 0.37 g anticancer drugs under stirring (150 rpm) and ultrasonication conditions, respectively.

### Synthesis of the Pt,Pd-NiO/SWCNTs Nanocomposite

1.0 g SWCNTs-COOH was dispersed in 100 mL distillated water solution under stirring conditions. Next, 0.182 g nickel nitrate hexahydrate + 0.016 g palladium dichloride and 0.016 g platinum(II) acetylacetonate were added to this solution, and stirring was continued for 30 min at 45°C. Afterward, 100 mL sodium hydroxide 0.2 M was added to the solution with no change in temperature or stirring speed. The obtained sample was dried in a vacuum oven at 100°C for 4 h. The black powder was then transferred into a furnace and calcinated for 4.0 h at 400°C.

### Preparation of Pt,Pd-NiO/SWCNTs/1B23DTFB/CP

The ratio of Pt,Pd-NiO/SWCNTs and 1B23DTFB in preparation of Pt,Pd-NiO/SWCNTs/1B23DTFB/CP were optimized in the presence of 500 μM daunorubicin (Figures S1, S2). Pt,Pd-NiO/SWCNTs/1B23DTFB/CP was developed by mixing carbon powder and Pt,Pd-NiO/SWCNTs as powder components in the ratio of 94:6 (w/w) and paraffin oil and 1B23DTFB as liquid binders in the ratio of 8:2 (v/v). The mixture was then carefully homogenized in an agate mortar using a pestle. The obtained paste was packed into a glass tube, and a copper wire was used for electrical contact.

### Real Sample Preparation

The injection and pharmaceutical serum samples were prepared from a local pharmacy and used as real samples for investigating the ability of Pt,Pd-NiO/SWCNTs/1B23DTFB/CP as a new analytical tool to determine daunorubicin and tamoxifen (Nolvadex). The samples were used directly and without any pretreatment. The standard addition method was selected as the analytical strategy for this goal.

## Results and Discussion

### Characterization of the Pt,Pd-NiO/SWCNTs Nanocomposite

The synthesized Pt,Pd-NiO/SWCNTs was characterized by different powerful methods, such as TEM and EDS. The recorded results relative to morphological investigation (TEM) is presented in Figure 1A. The decorated nanoparticle on the surface of the SWCNTs is clearly shown in the TEM image. The particle size of about 10 nm was estimated for the Pt,Pd-NiO nanoparticle decorated on the surface of the SWCNTs. Figure 1B (EDS analysis data) successfully confirms the presence of Pt, Pd, Ni, and O, C elements in the Pt,Pd-NiO/SWCNTs structure, which approves high purity in the synthesis procedure.

**Figure 1:** **(A)** TEM and **(B)** EDS images of Pt,Pd-NiO/SWCNT nanocomposites.

### Electrochemical Behavior of Daunorubicin

The I–V response of daunorubicin was recorded in different pH (pH range 5.0–9.0) values in order to study the effect of proton concentration in the current and potential of the anticancer drug (Figure 2 inset). The plot of E vs. pH showed a linear relation with equation E_pa_ = 0.061 pH + 1.049 (*R*^2^ = 0.998) on the surface of Pt,Pd-NiO/SWCNTs/1B23DTFB/CP as an electrochemical sensor. This value of slope (0.061) confirmed equal electron and proton values in the redox reaction of daunorubicin on the surface of Pt,Pd-NiO/SWCNTs/1B23DTFB/CP (Figure 2). In comparing oxidation signals (I–V curves), the best oxidation signal was observed at pH = 7.0 (Figure S3). Therefore, pH = 7.0 can be selected as the best electrochemical condition for the analysis of daunorubicin.

**Figure 2:** E-pH plot relative to electro-oxidation of 200 μM daunorubicin at the surface of Pt,Pd-NiO/SWCNTs/1B23DTFB/CP (*n* = 4). (Inset) I–V curves of 200 μM daunorubicin at the surface of Pt,Pd-NiO/SWCNTs/1B23DTFB/CP in the pH range 5.0–9.0.

### Role of Pt,Pd-NiO/SWCNTs and 1B23DTFB in the Prepared Sensor

The role of Pt,Pd-NiO/SWCNTs and 1B23DTFB in the fabrication of Pt,Pd-NiO/SWCNTs/1B23DTFB/CP and their effects on the oxidation signal of daunorubicin were investigated by the I–V method. As can be seen, daunorubicin showed a weak oxidation signal with a current of 7.74 μA and potential of 720 mV on the surface of the carbon paste electrode (Figure 3, Curve a). After modification of the CPE with the Pt,Pd-NiO/SWCNTs nanocomposite, the oxidation current of daunorubicin improved to 40.25 μA, and the oxidation potential of daunorubicin was decreased to 680 mV (Figure 3, Curve b). Under the same conditions and after modification of the CPE with 1B23DTFB as a binder, the oxidation current of daunorubicin was improved to 50.35 μA, and the oxidation potential of daunorubicin was decreased to 670 mV (Figure 3, Curve c). These improvements in the redox reaction of daunorubicin by Pt,Pd-NiO/SWCNTs and 1B23DTFB are correlated with the good electrical conductivity of the mediators. Therefore, the modification of CPE with Pt,Pd-NiO/SWCNTs and 1B23DTFB and making Pt,Pd-NiO/SWCNTs/1B23DTFB/CP a highly conductive sensor were selected. On the surface of the Pt,Pd-NiO/SWCNTs/1B23DTFB/CP, the oxidation current of daunorubicin was about 76.04 μA, and the oxidation potential of daunorubicin was decreased to 610 mV (Figure 3, curve d). Comparing the oxidation signal of daunorubicin on the surface of CPE with Pt,Pd-NiO/SWCNTs/1B23DTFB/CP revealed a 9.8-times increase in current and a decrease of about 110 mV in the oxidation potential of the drug. The effects of Pt,Pd-NiO/SWCNTs and 1B23DTFB on improving conductivity of the sensor were investigated by recording current density data. For this goal and in the first step, the active surface areas of the CPE, Pt,Pd-NiO/SWCNTs/CP, 1B23DTFB/CP, and Pt,Pd-NiO/SWCNTs/1B23DTFB/CP were calculated to be about 0.13, 0.19, 0.2, and 0.22 cm^2^, respectively. Using active surface area data and the oxidation current of daunorubicin on the surface of different electrodes, the current density data was drawn and is shown in the inset of Figure 3. The diagrams confirm the improved conductivity of CPE after modification with Pt,Pd-NiO/SWCNTs nanocomposite and 1B23DTFB.

**Figure 3:** Cyclic voltammograms 500 μM daunorubicin at surface of (a) CPE; (b) Pt,Pd-NiO/SWCNTs/CP; (c) B23DTFB/CP; and (d) Pt,Pd-NiO/SWCNTs/1B23DTFB/CP. (Inset) Current density data relative electro-oxidation of 500 μM daunorubicin at surface of different electrodes.

The I–V signals of 100 μM daunorubicin on the surface of Pt,Pd-NiO/SWCNTs/1B23DTFB/CP and in the scan rate range of 10–450 mV/s were recorded under optimum conditions (Figure 4 inset). The results of the relationship between the current of daunorubicin and ν^1/2^ on the surface of Pt,Pd-NiO/SWCNTs/1B23DTFB/CP are shown in Figure 4. The equation I_pa_ = 1.9238 ν^1/2^ – 4.1438 (*R*^2^ = 0.9942) was recorded for this study. This equation and the linear relation between current and ν^1/2^ on the surface of Pt,Pd-NiO/SWCNTs/1B23DTFB/CP suggest that the electro-oxidation of daunorubicin is under the diffusion control.

**Figure 4:** I-ν^1/2^ plot relative to electro-oxidation of 100 μM daunorubicin at surface of Pt,Pd-NiO/SWCNTs/1B23DTFB/CP (*n* = 4). (Inset) Cyclic voltammograms of 100 μM daunorubicin at the surface of Pt,Pd-NiO/SWCNTs/1B23DTFB/CP at scan rates (a) 10.0; (b) 20.0; (c) 40.0; (d) 100.0; (e) 150.0; (f) 200.0; (g) 350.0; and (h) 450.0 mV/s.

Figure 5 shows the Tafel plot relative to oxidation of 100 μM daunorubicin at the surface of Pt,Pd-NiO/SWCNTs/1B23DTFB/CP. Using the slope of the Tafel plot, the value of α was calculated 0.8.

**Figure 5:** Tafel plot for Pt,Pd-NiO/SWCNTs/1B23DTFB/CP with a scan rate of 10 mV/s in the presence of 100 μM daunorubicin.

With the confirmation of the diffusion process during the daunorubicin oxidation process on the surface of Pt,Pd-NiO/SWCNTs/1B23DTFB/CP, the chronoamperometric method with applied potential of 750 mV was used to determine the diffusion coefficient (D) of daunorubicin (Figure 6). The inset in Figure 6 shows the Cottrell plots relative to daunorubicin oxidation on the surface of Pt,Pd-NiO/SWCNTs/1B23DTFB/CP. Using the obtained slopes relative to daunorubicin oxidation in the different concentration ranges and on the surface of Pt,Pd-NiO/SWCNTs/1B23DTFB/CP, the value of D was calculated to be about 1.43 × 10^−5^ cm^2^/s.

**Figure 6:** **(A)** Chronoamperograms obtained at Pt,Pd-NiO/SWCNTs/1B23DTFB/CP in the solution containing (a) 400, (b) 500, and (c) 600 μM daunorubicin. **(B)** Cottrell plots obtained from chronoamperogram signals.

### Stability Investigation of Pt,Pd-NiO/SWCNTs/1B23DTFB/CP

The storage stability of Pt,Pd-NiO/SWCNTs/1B23DTFB/CP was investigated by storing the amplified daunorubicin sensor for 40 days. The Pt,Pd-NiO/SWCNTs/1B23DTFB/CP had maintained 90.0% of its initial current in the presence of 500 μM daunorubicin after 1 month; after this time, the current was drastically reduced, which confirmed that Pt,Pd-NiO/SWCNTs/1B23DTFB/CP had the ability to efficiently and analytically measure daunorubicin (Figure S4).

### Analytical Approach for the Simultaneous Determination of Daunorubicin in the Presence of Tamoxifen

According to previous reports, daunorubicin and tamoxifen may be present simultaneously in biological solutions. Accordingly, the Pt,Pd-NiO/SWCNTs/1B23DTFB/CP's ability to determine these two anticancer drugs was examined. The differential pulse voltammograms (DPVs) of daunorubicin were recorded on the surface of Pt,Pd-NiO/SWCNTs/1B23DTFB/CP, and a linear relation between current and daunorubicin concentration was observed in the range of 0.008–350 μM with equation I_pa_ = 0.2351 C_daunorubicin_ + 2.7029 (*R*^2^ = 0.9954) (Figure S5). The differential pulse voltammograms of tamoxifen were also recorded on the surface of Pt,Pd-NiO/SWCNTs/1B23DTFB/CP, and a linear relation between current and tamoxifen concentration was observed in the range of 0.5–330 μM with equation I_pa_ = 0.4178 C_tamoxifen_ + 0.0867 (*R*^2^ = 0.9983) (Figure S6). Pt,Pd-NiO/SWCNTs/1B23DTFB/CP showed detection limits of 3.0 nM and 0.1 μM for daunorubicin and tamoxifen, respectively.

The DP voltammograms of the solutions containing different concentrations of daunorubicin+ tamoxifen were recorded on the surface of Pt,Pd-NiO/SWCNTs/1B23DTFB/CP (Figure 7A). The plots of current vs. concentration of daunorubicin or tamoxifen (for this study) are presented in Figures 7B,C. The results for the slopes presented in Figures 7A,B are quite similar to the results for separate drug analyses. As an example, the investigation of the linear dynamic range for daunorubicin alone showed a slope of 0.2351 μA/μM. This value of sensitivity is very close to the recorded sensitivity in simultaneous analyses (0.2267 μA/μM). Two separated oxidation signals were observed in the solutions containing different concentrations of daunorubicin + tamoxifen with ΔE = 315 mV. These results confirm the powerful and selective ability of Pt,Pd-NiO/SWCNTs/1B23DTFB/CP as an electroanalytical sensor for the determination of daunorubicin in the presence of tamoxifen.

**Figure 7:** **(A)** DPVs of Pt,Pd-NiO/SWCNTs/1B23DTFB/CP containing different concentrations of daunorubicin-tamoxifen (from inner to outer vs. μM): 35.0 + 20.0; 50.0 + 30.0; 75.0 + 45.0; 100.0 + 55.0; 140.0 +75.0 and 180.0 + 90.0, respectively. Insets: Plots of I_p_ vs. **(B)** daunorubicin and **(C)** tamoxifen concentrations (*n* = 4).

### Real Sample and Interference Studies

The selectivity of Pt,Pd-NiO/SWCNTs/1B23DTFB/CP for the determination of daunorubicin was investigated in this step. The results are presented in Table S1 and confirm the selectivity of Pt,Pd-NiO/SWCNTs/1B23DTFB/CP as a new electroanalytical sensor for the determination of daunorubicin.

In the final step, the ability of Pt,Pd-NiO/SWCNTs/1B23DTFB/CP to determine daunorubicin in different real samples, such as injection and pharmaceutical serums, was checked using the standard addition method. A recovery rate of 96.86–102.25% was detected, confirming the high capability of Pt,Pd-NiO/SWCNTs/1B23DTFB/CP in determining daunorubicin and tamoxifen in real samples (Table 1).

**Table 1:** Determination of daunorubicin and tamoxifen in real samples (*n* = 4).

**Samples**	**Daunorubicin added (μM)**	**Tamoxifen added (μM)**	**Founded of daunorubicin (μM)**	**Founded of tamoxifen (μM)**	**Recovery % of daunorubicin**	**Recovery% of tamoxifen**
Injection samples of daunorubicin	—	—	2.04 ± 0.11	—	—	—
	5.00	—	7.08 ± 0.21	—	100.5	—
Dextrose saline	—	—	< LOD	< LOD	—	—
	35.00	20.00	34.79 ± 0.66	20.54 ± 0.63	99.4	102.25
Injection samples of tamoxifen	—	—	—	5.11 ± 0.34	—	—
	—	5.00	—	4.95 ± 0.76	—	96.86

## Conclusion

In this study, Pt,Pd-NiO/SWCNTs were synthesized using the one-pot procedure and combining chemical precipitation and ultrasonic sonochemical deposition methods. The characterization data confirmed the good purity and distribution for the synthesized nanocomposite, which also showed the improved conductivity effect of the fabricated sensor for the determination of daunorubicin. It is noteworthy that the designed sensor can well measure daunorubicin in the presence of tamoxifen (two breast anticancer drugs with a ΔE = 315 mV. Pt,Pd-NiO/SWCNTs/1B23DTFB/CP showed a good ability for determining daunorubicin and tamoxifen with detection limits of 3.0 nM and 0.1 μM, respectively. Pt,Pd-NiO/SWCNTs/1B23DTFB/CP also showed a recovery range of 96.86–102.25% for the analyses of daunorubicin and tamoxifen, confirming the high capacity of the fabricated sensor for the real sample analysis of anticancer drugs.

## Data Availability Statement

All datasets presented in this study are included in the article/Supplementary Material.

## Author Contributions

MA: experimental part as a Ph.D. student. PA and SM: introduce thesis and work as supervisor. HK-M and A-MT: write the paper and advisor of work. All authors contributed to the article and approved the submitted version.

## Conflict of Interest

The authors declare that the research was conducted in the absence of any commercial or financial relationships that could be construed as a potential conflict of interest. The reviewer FK declared a past co-authorship with one of the authors HK-M to the handling editor.
